The article "The Anesthetic Effect and Safety of Dexmedetomidine in Cesarean Section: A Meta-Analysis" was retracted in 2023. Reasons: suspected computer-generated content; unreliable results or conclusions; lack of ethics approval or compliance; missing or withdrawn patient consent.

# The Anesthetic Effect and Safety of Dexmedetomidine in Cesarean Section: A Meta-Analysis

**DOI:** 10.1155/2022/1681803

**Published:** 2022-05-14

**Authors:** Gang Pang, Yuanmao Zhu, Yan Zhou, Shanshan Tong

**Affiliations:** ^1^Department of Anesthesiology, Chongqing University Jiangjin Hospital, School of Medicine, Chongqing University, Chongqing, China; ^2^Department of Painology, Chongqing University Jiangjin Hospital, School of Medicine, Chongqing University, Chongqing, China; ^3^Department of Obstetrics and Gynecology, Chongqing University Jiangjin Hospital, School of Medicine, Chongqing University, Chongqing, China

## Abstract

**Objective:**

To evaluate the anesthetic effect and safety of dexmedetomidine in cesarean section.

**Methods:**

The Cochrane Library, EMBASE, and PubMed databases (established until September 2020) were searched by computer. Two authors independently screened and extracted literature related to the application of dexmedetomidine in the cesarean section according to inclusion and exclusion criteria. The control group received either subarachnoid block (lumbar anesthesia) or combined lumbar anesthesia and epidural anesthesia (combined lumbar epidural anesthesia) with bupivacaine or combined bupivacaine and fentanyl. The observation group was additionally given dexmedetomidine based on the control group, to analyze the anesthetic effect and safety of dexmedetomidine in cesarean section.

**Results:**

A total of 580 cesarean delivery women were included in 8 studies, and the results showed that the peak time of sensory block in the observation group was shorter than that in the control group (standard mean difference = −0.28; 95% confidence interval: -0.48, -0.08; *P* = 0.006), sensory block lasted longer than that in the control group (standard mean difference = 1.49; 95% confidence interval: 1.21, 1.78; *P* < 0.00001), the sedation rate was higher than that in the control group, the onset of the first postoperative pain was significantly delayed compared with that in the control group, and the incidence of postoperative pain, nausea and vomiting, postoperative chills, and fever was lower than that in the control group (*P* < 0.05).

**Conclusion:**

Dexmedetomidine combined with lumbar anesthesia or combined lumbar epidural anesthesia for women in cesarean section has more clinical benefits and better safety.

## 1. Introduction

Cesarean section is a relatively common surgical method in clinical practice [1]. After a cesarean section, women are generally accompanied by strong incision pain and uterine involution pain, which not only affects their postoperative recovery but also leads to a sympathetic nervous response in patients, thereby promoting the secretion of catecholamines which inhibits the release of prolactin, which in turn affects lactation [2], which in turn affects the growth and development of neonates [3]. Therefore, perfect analgesia must be given after cesarean section. At present, the most ideal analgesia after cesarean section not only needs to achieve effective analgesia but also must minimize the impact on mother and baby [4].

The choice of anesthesia methods and anesthetic drugs has a great influence on the recovery of cesarean section women. Subarachnoid block (spinal anesthesia) or combined spinal-epidural anesthesia (spinal-epidural anesthesia) has a precise analgesic effect. It has the advantages of complete nerve block and is widely used in the cesarean section [5]. The duration of analgesia after spinal anesthesia is short, and patients after cesarean section spinal anesthesia often experience visceral pain, nausea, vomiting, and other adverse reactions [6]. Although bupivacaine can prolong the sensory and motor block time, the postoperative analgesic effect is still unsatisfactory. Therefore, adjuvant analgesic and sedative drugs are often added to the spinal anesthesia to prolong the postoperative analgesic effect [7]. Combined spinal-epidural anesthesia is often added with adjuvant drugs to improve postoperative analgesia and promote early ambulation; at the same time, adjuvant drugs reduce the dose of bupivacaine, which can reduce the occurrence of adverse reactions after anesthesia [8]. Fentanyl can be used as an adjuvant drug for spinal anesthesia to prolong postoperative analgesia. It has the characteristics of fast peaking, a strong analgesic effect, and a short half-life. It is widely used in postoperative intravenous analgesia, but it can cause many adverse reactions, such as nausea, vomiting, urinary retention, and respiratory depression [9]. At the same time, maternal anxiety, chills, nausea, and vomiting are prone to adverse reactions during cesarean section [10]. Studies have shown that intraoperative use of a certain dose of dexmedetomidine (intravenous infusion started after the fetus is born) to assist sedation can prevent the onset of chills and significantly reduce maternal uterine contraction due to drugs [11]. The incidence of adverse reactions such as nausea and vomiting caused by the use of the puerperium and the surgical traction reaction is conducive to maintaining the stability of the intraoperative circulation and does not affect breathing, while the puerperal has stable breathing and circulation [12]. It will be beneficial to the blood perfusion of important organs such as the heart, brain, and kidney and produce a certain organ protection effect, which will help improve the safety and comfort of the mother during the operation [13]. Dexmedetomidine is a novel highly selective adrenergic receptor agonist, which is a selective adrenergic *α*2 receptor agonist. With its high selectivity and high efficacy, dexmedetomidine has great advantages in analgesia and sedation, and its hemodynamic stability can be used as an adjunct to spinal anesthesia [14, 15]. A large number of studies have also shown that fentanyl/bupivacaine combined with dexmedetomidine for intravenous analgesia after cesarean section can enhance the analgesic effect, reduce the number of analgesic drugs, and reduce the incidence of drug-related adverse reactions, to improve patient satisfaction [16, 17]. However, there is still a lack of clear evidence on the anesthesia effect and safety of dexmedetomidine in cesarean section of the parturient.

## 2. Materials and Methods

### 2.1. Inclusion and Exclusion Criteria

Inclusion criteria: randomized controlled trial with full English text. Included patients were adults (>18 years old), cesarean delivery women, American Society of Anesthesiologists (ASA) rating I~III. Interventions: the control group used bupivacaine or bupivacaine combined with fentanyl for lumbar anesthesia or combined lumbar epidural anesthesia. The observation group was additionally given dexmedetomidine based on the control group. Outcome indicators: onset time of the sensory block, the peak time of sensory block plane, duration of sensory block, recovery time of motor block; intraoperative sedation; postoperative pain (time of first postoperative pain attack, postoperative pain occurrence rate); incidence of adverse reactions (hypotension, bradycardia, nausea and vomiting, pruritus, dizziness, intraoperative pain, urinary retention, chills, fever, diarrhea, and headache). Exclusion criteria: nonrandomized controlled trials such as conference abstracts, case reports, case series, and retrospective studies; women with pregnancy complications. Nonspinous or combined spinal-epidural anesthesia. Outcome indicators were not met.

### 2.2. Literature Retrieval

Cochrane Library, EMBASE, and PubMed databases (established until September 2021) were searched by computer using a combination of text words and mesh terms, including “detomidine” and “Cesarean section”.

### 2.3. Literature Screening and Data Extraction

In strict accordance with the Cochrane Handbook standard, two authors independently screened the literature and extracted data according to the inclusion and exclusion criteria.

The inclusion criteria of this study are ① the research object must be adults; ② the grouping of the experimental group and the control group is clear; ③ baseline characteristics of subjects are included (e.g., age, ASA rating, whether multiple pregnancies, medication methods, and additional medications).

Literature exclusion criteria: ① non-English literature; ② literature types that cannot provide specific data such as review, letter, case report, and abstract; ③ incomplete literature data and repeated literature data; ④ serious defects in literature design, no control group experiment, and no clear diagnostic criteria for the experimental group; ⑤ studies without any control group; ⑥ full version of text missing; and ⑦ no clear outcome.

### 2.4. Literature Quality Evaluation

The methodological quality of the included randomized controlled trials was assessed using the risk of bias assessment tool provided by the Cochrane Handbook [6]. The evaluation contents of each included study included ① random sequence generation, ② allocation concealment, ③ implementer and participant blinding, ④ outcome assessor blinding, and ⑤ incomplete data reporting, other sources of bias.

### 2.5. Statistical Analysis

The dichotomous variable effect index was expressed by relative risk (RR) and its 95% confidence interval (95% CI); the continuous variable effect index was expressed by standard mean difference (SMD) and its 95% CI. Heterogeneity was quantified using *I*^2^ and *X*^2^ tests. *I*^2^ ≥ 50%, *P* < 0.1 indicates statistical heterogeneity, and the source of heterogeneity should be sought at this time. Sensitivity analysis can be used when necessary to test the stability of the results. If *I*^2^ < 50%, *P* < 0.1, indicating that there is no heterogeneity among the studies, a fixed effect model was used for analysis. *P* < 0.05 means the difference is statistically significant.

## 3. Results

### 3.1. Literature Screening Results

A total of 314 articles were retrieved, 211 articles remained after excluding duplicate articles, 21 articles remained after preliminary screening of reading titles and abstracts, 13 articles were excluded after full-text reading, and the remaining 8 articles were included in the study.

### 3.2. Basic Characteristic of the Included Literature

Eight studies with a total of 580 cesarean sections were included in this study (Figure 1). The characteristics of the included literature are listed in Table 1.

### 3.3. Risk of Bias Assessment

Figure 2 shows that the included studies have varying degrees of risk of bias.

### 3.4. Anesthesia Blocking Effect

Six studies [18, 19, 22–25] reported the time to peak sensory block level. There was no significant heterogeneity among the studies (*P* = 0.94, *I*^2^ = 0%), and the fixed effect model was used for analysis. The results showed that the peak time of the sensory block plane in the observation group was shorter than that in the control group (SMD = −0.28; 95% CI: -0.48, -0.08; *P* = 0.006) (Figure 3). Four studies [19, 22, 24, 25] reported duration of sensory block. There was no significant heterogeneity among the studies (*P* = 0.49, *I*^2^ = 0%), and the fixed effect model was used for analysis, and the results showed that the duration of sensory block in the observation group was longer than that in the control group (SMD = 1.49, 95% CI: 1.21-1.78, *P* < 0.001) (Figure 4). Six studies [18, 19, 22–25] reported motor block recovery time. There was significant heterogeneity among the studies (*P* < 0.001, *I*^2^ = 89%), and the results showed that the recovery time of motor block between the two groups was statistically significant (SMD = 0.71; 95% CI: 0.11, 1.42; *P* = 0.02) (Figure 5).

### 3.5. Sedation

Three studies [18, 23, 25] reported on intraoperative sedation. There was no significant heterogeneity among the studies (*P* = 0.17, *I*^2^ = 47%), and the fixed effect model was used for analysis, and the results showed that the sedation rate in the observation group was higher than that in the control group (RR = 1.61; 95% CI: 1.23, 2.10; *P* < 0.001) (Figure 6).

### 3.6. Postoperative Analgesia

Five studies [18, 19, 22, 24, 25] reported the time to the first postoperative pain attack. There was significant heterogeneity among the studies (*P* < 0.001, *I*^2^ = 96%). The random effects model was used for analysis. The results showed that the first postoperative pain attack time in the observation group was significantly delayed compared with the control group (SMD = 4.68, 95% CI: 2.26-7.10, *P* < 0.001) (Figure 7). One study [18] reported the incidence of postoperative pain, and the results showed that the incidence of postoperative pain in the observation group was significantly lower than that in the control group (*R* = 0.25, 95% CI: 0.08 -0.78, *P* = 0.02).

### 3.7. Adverse Reactions

Eight studies reported the incidence of postoperative adverse reactions. The results showed that the incidence of nausea and vomiting, postoperative chills, and fever in the observation group was lower than that in the control group (*P* < 0.05). Other adverse reactions in the two groups were hypotension, bradycardia, and itching. There was no significant difference in the incidences of dizziness, intraoperative pain, urinary retention, diarrhea, and headache (*P* > 0.05) (Table 2).

### 3.8. Publication Bias

Funnel plot analysis was conducted on 8 articles reporting hypotension, and the results showed that the funnel plot was symmetric, so the bias was not obvious (Figure 8).

## 4. Discussion

For cesarean section anesthesia, subarachnoid or epidural injection of local anesthetics such as bupivacaine or ropivacaine or opioids is often the option of choice [5]. On this basis, adjuvant systemic sedative drugs may help to improve the effect of anesthesia and reduce the occurrence of adverse reactions [26]. Dexmedetomidine is an auxiliary sedative commonly used in clinical practice and is also widely used in cesarean section anesthesia. However, the effects of dexmedetomidine on the anesthetic effect and adverse reactions of the cesarean section under lumbar anesthesia or combined lumbar epidural anesthesia have not been determined [27, 28]. This meta-analysis showed that intravenous dexmedetomidine-assisted sedation based on lumbar anesthesia or combined lumbar epidural anesthesia could achieve better analgesic and sedative effects. Dexmedetomidine can shorten the peak time and prolong the duration of the sensory block. It can significantly delay the onset of the first postoperative pain and reduce the incidence of postoperative pain. In addition, the incidence of hypotension and bradycardia did not increase after the addition of dexmedetomidine, indicating that it did not lead to instability in hemodynamics. But it reduced the incidence of nausea, vomiting, chills, and fever. The risk bias of included studies in this system evaluation is low, and selection bias may affect the results of the study.

Dexmedetomidine has the advantages of sensory block and analgesia. On the one hand, due to its effect at the spinal cord level, it inhibits the release of norepinephrine and blocks the transmission of pain signals to the brain by acting on A2 receptors in the presynaptic membrane and posterior membrane of the spinal cord [29]. On the other hand, due to its effect on the A2 receptor of the cerebral vena cava, it inhibits the excitation of the neurons in the vena cava and blocks the pain nerve signal transduction pathway of the medullary globus-spinal cord to achieve sedation and analgesia [30]. Studies have found that in patients undergoing abdominal and lower limb surgery, epidural anesthesia with dexmedetomidine shortens the onset time of sensory block and prolongs postoperative analgesia time. Some studies have also proved that the analgesic effect of dexmedetomidine is superior to clonidine in vaginal hysterectomy or children's lower abdominal surgery [31–33]. By acting on the central nervous system, dexmedetomidine can affect the activities of sympathetic and parasympathetic nerves, accelerate gastrointestinal empties and peristalsis, reduce the stimulation of the gastrointestinal tract stretch to the vomiting center, and thus reduce the incidence of nausea and vomiting. Dexmedetomidine inhibits the central temperature regulation system and reduces the perioperative stress response caused by elevated adrenaline, thus reducing the occurrence of chills [34, 35].

The advantage of this study lies in the systematic retrieval of relevant literature, two-person literature screening, and data extraction, which reduces the systematic error in the operation process. At the same time, the risk of bias in the included literature was low, and the meta-analysis had good homogeneity, so the results were relatively reliable. The shortcoming of the study is that due to the few kinds of research in related fields and the small sample size, the results may be inaccurate, thus affecting the real effect of the results. Therefore, the systematic evaluation shows that dexmedetomidine can bring more clinical benefits to patients based on lumbar anesthesia or combined lumbar epidural anesthesia. However, due to the small sample size, clinicians should be cautious in this conclusion. At present, there are few studies in this field, and it is urgent to confirm with a large sample of randomized controlled trials.

## 5. Conclusion

Dexmedetomidine combined with lumbar anesthesia or combined lumbar epidural anesthesia for women in cesarean section has more clinical benefits and better safety.

## Figures and Tables

**Figure 1:** PRISMA flowchart of the included studies.

**Figure 2:** Risk of bias summary of the included studies.

**Figure 3:** Forest plot of the peak time of sensory block plane.

**Figure 4:** Forest plot of duration of sensory block.

**Figure 5:** Forest plot of recovery of motor block.

**Figure 6:** Forest plot of sedation rate.

**Figure 7:** Forest plot of time to first analgesics.

**Figure 8:** Funnel plot analysis of 8 articles reporting hypotension.

**Table 1:** The basic characteristic of the included literature.

Study (year)	Age (years, *x* ± *s*)	Operation time (min, *x* ± *s*)	Experimental group (*n*)	Control group (*n*)
Hanoura (2013) [18]	29.8 ± 4.6	49 ± 8	2 ml of spinal anesthesia 0.5% bupivacaine+10 ml of epidural injection 0.25% bupivacaine+dexmedetomidine 1 *μ*/kg and fentanyl 100 *μ*g (*n* = 25)	2 ml of lumbar anesthesia 0.5% bupivacaine+10 ml of epidural injection 0.25% bupivacaine+fentanyl 100 *μ*g (25)
Li (2015) [19]	30.30 ± 3.81	45.89 ± 8.95	Lumbar anesthesia 10 mg bupivacaine+10 *μ*g dexmedetomidine (21)	Lumbar anesthesia 10 mg bupivacaine (21)
Liu (2015) [20]	31 ± 5	39.1 ± 6.3	1.5 ml of lumbar anesthesia 0.5% bupivacaine+0.5 *μ*g/kg dexmedetomidine (40); 1.5 ml of lumbar anesthesia 0.5% bupivacaine+1 *μ*/kg dexmedetomidine (40) (*n* = 80)	1.5 ml of lumbar anesthesia 0.5% bupivacaine+20 ml of 0.9% sodium chloride injection (*n* = 40)
Nasseri (2017) [21]	32.16 ± 5.24	51.04 ± 19.39	Lumbar anesthesia 12.5 mg 0.5% bupivacaine+5 *μ*g dexmedetomidine (25)	Lumbar anesthesia 12.5 mg 0.5% bupivacaine+0.5 ml of 0.9% sodium chloride injection (25)
Sun (2015) [22]	29.75 ± 4.90	42.89 ± 9.25	2 ml of lumbar anesthesia 0.5% bupivacaine+10 *μ*g dexmedetomidine (30)	2 ml of lumbar anesthesia 0.5% bupivacaine+1.0 ml of 0.9% sodium chloride injection (30)
Yousef (2015) [23]	28.5 ± 5.7	50.4 ± 4.9	1.5 ml of spinal anesthesia 0.5% bupivacaine+10 ml of epidural infusion 0.25% bupivacaine+1 ml of dexmedetomidine 0.5 WG/kg+1 ml of fentanyl 50 *μ*g (40)	1.5 ml of spinal anesthesia 0.5% bupivacaine+10 ml of epidural injection 0.25% bupivacaine+1 ml of 0.9% sodium chloride injection+1 ml of fentanyl 50 *μ*g (40)
Qi (2016) [24]	29.75 ± 3.87	39.46 ± 7.81	2 ml of 0.5% bupivacaine containing 5 *μ*g of dexmedetomidine (*n* = 40)	2 ml of 0.5% bupivacaine alone (*n* = 40)
Xia (2018) [25]	25.5 ± 3.5	45 ± 7.5	Bupivacaine+5 mcg dexmedetomidine (45)	Bupivacaine+the same volume of saline (45)

**Table 2:** Meta-analysis of adverse reactions after cesarean section between two groups.

Outcomes	Sample size	RR (95% CI)	*P* value
Hypotension [18–25]	580	0.89 (0.70~1.14)	0.36
Bradycardia [18, 19, 21–24]	360	1.48 (0.70~3.12)	0.31
Nausea and vomiting [18–25]	580	0.74 (0.57~0.96)	0.03
Pruritus [18, 19, 22–25]	400	1.00 (0.35~2.89)	1
Dizziness [18, 23]	130	2.00 (0.19~21.18)	0.56
Postoperative pain [18]	50	0.08 (0.00~1.30)	0.08
Urine retention [19]	42	5.00 (0.25~98.27)	0.29
Shivering [18, 21, 22, 24, 25]	328	0.40 (0.24~0.65)	0.0003
Fever [20]	120	0.05 (0.00~0.81)	0.04
Diarrhea [20]	120	0.75 (0.13~4.31)	0.75
Headache [20]	120	0.17 (0.01~4.05)	0.27

## Data Availability

The data used to support this study are available from the corresponding author upon request.
